The article "Application and Optimization of Luenberger Observer Phase-Locked Loop and Inductance-Free Vector Control Method for Aviation Three-Phase Converter in Wearable Equipment" was published in 2022. Journal: Comput Intell Neurosci.

# Application and Optimization of Luenberger Observer Phase-Locked Loop and Inductance-Free Vector Control Method for Aviation Three-Phase Converter in Wearable Equipment

**DOI:** 10.1155/2022/9480125

**Published:** 2022-08-13

**Authors:** Bo Zeng, Yuxiang Sun

**Affiliations:** ^1^College of Automation Engineering, Nanjing University of Aeronautics and Astronautics, Nanjing 211106, China; ^2^School of Management & Engineering, Nanjing University, Nanjing 210093, China; ^3^School of Computing and Engineering, University of Derby, Derby DE22 1GB, UK

## Abstract

This work aims to strengthen the comprehensive performance of the Luenberger observer in the application of aviation three-phase converter and in physical exercise wearable devices to effectively detect human physiological signals. Firstly, the use status and characteristics of three-phase converters are discussed. Then, the Luenberger observer and its optimization process are described. Finally, the Luenberger observer is optimized through phase-locked loop technology and the vector control method. The experimental results indicate that the PLL of the steady-state linear Kalman filter is applicable to the multielectric aircraft converter for the aviation variable frequency power supply. The phase-locked loop of the steady-state linear Kalman filter is complicated, and the output angular frequency is inconsistent with the angular frequency of the actual voltage of the aircraft variable-frequency power supply. Consequently, it does not have the function of frequency locking. On the contrary, the Luenberger observer phase-locked loop designed here is suitable for the multielectric aircraft converter for the aircraft variable-frequency power supply. In addition, it is simpler than the steady-state linear Kalman filter phase-locked loop and realizes the frequency-locking function. In addition, the vector control method significantly improves the control performance of the Luenberger observer. The control error of the original observer is about 0.24°, and the control error of the optimized observer is about 0.18°. This work provides technical support for the performance optimization of the Luenberger observer and contributes to the performance improvement of the aviation three-phase converter.

## 1. Introduction

With the advance of society, sports have developed into a mainstream project in society. It is of great significance to effectively detect human physiological functions and control the state of human movement during physical exercise. At the same time, the capacity and power generation efficiency of the aircraft power system have been continuously improved with the development of multielectric aircraft technology. The advantages of aviation variable frequency power supply without the need to continuously install converters have gradually emerged [1]. Three-phase converters, especially three-phase rectifiers, are crucial power conversion links in airborne electrical equipment. The high power factor is the main indicator to measure the performance of an aviation rectifier [2]. It is necessary to obtain grid voltage phase information, which is usually done by a phase-locked link, to achieve high power factor operation of the rectifier [3, 4]. It is also important to optimize the Luenberger observer by vector control, as it is the central bearing system of the phase-locked loop. Applying the Luenberger observer in sports can improve people's exercise efficiency by monitoring the physiological function of the human body under exercise conditions. This design has breakthrough significance and provides a significant reference for the development of sports. Many studies have provided technical support for this developing research.

Sun et al. reported that the current permanent magnet synchronous motor has been widely used in many fields, such as vehicles, air conditioners, refrigerators, and fans, because of its high power density, torque inertia ratio, simple structure, and fast dynamic response. With the continuous expansion of application fields, the high-performance permanent magnet synchronous motor control strategy has become the focus of attention and the mainstream control strategy. The key of the permanent magnet synchronous motor vector control method is to obtain the motor speed and rotor position. However, installing and maintaining the traditional mechanical sensor is challenging, increasing the system cost and mechanical structure complexity and reducing the system reliability. Therefore, the sensorless control of permanent magnet synchronous motor has become a significant development trend in the future [5]. Weichbold et al. proposed a real-time detection method of demagnetization fault based on state observer, aimed at the problem of demagnetization of permanent magnet synchronous motor. They also established a mathematical model of the demagnetization fault of the built-in permanent magnet synchronous motor by selecting the stator current in the magnetic field synchronous rotating coordinate system as the state variable. Then, two observers were used to estimate the permanent magnet flux linkage in real-time. Firstly, the Luenberger observer was used to isolate the influence of motor speed change on the observer error equation in the system matrix. Then, the sliding mode variable structure observer was designed. Besides, the formula for estimating the flux linkage of the permanent magnet was established according to the equivalent control principle of the sliding mode variable structure. A continuous function instead of a symbolic function was used to construct the loss of excitation fault reconstruction algorithm to reduce the jitter of the sliding mode motion. Finally, the feasibility and effectiveness of the proposed method were proved by simulation [6]. Tokić et al. (2021) stated that a permanent magnet synchronous motor has the advantages of small volume, small inertia, and light weight, so it is increasingly widely used in various fields. At present, vector control and direct torque control are most used in various control algorithms of permanent magnet synchronous motors. These two control methods both need a rotor position sensor, limiting the application range of the system. The existing speed sensorless control strategy of permanent magnet synchronous motors is mainly divided into the high-speed back electromotive force (EMF) estimation method and the low-speed rotor salient pole tracking method. The high-frequency rotating voltage injection method is widely used for salient pole tracking. It can estimate the rotor's position by injecting a high-frequency rotating voltage vector and processing a high-frequency current [7]. Feng et al. (2020) designed an improved feedback gain matrix based on the Luenberger observer to apply the high-quality vector control of speed sensorless to variable frequency all-in-one machine. This matrix can ensure the convergence speed of rotor flux observation and speed estimation and simultaneously ensure the stability of motor speed observation in the low-frequency region. Besides, an adaptive resonance controller was designed to solve motor terminal current resonance caused by bus voltage fluctuation under large load conditions. The compensation amount of the resonant regulator was adjusted in real-time through the amplitude value of the harmonic wave in the motor end current. This operation can realize the no static error control and good dynamic performance of the harmonic wave of a specific frequency in the motor end current. Simulation and motor drag experiments verified the effectiveness of the control strategy [8].

To sum up, this work first discusses the current situation and characteristics of the three-phase converter. Then, the principle and characteristics of the Luenberger observer are explored. Finally, the vector control method of the Luenberger observer is optimized to design a phase-locked loop. The innovation of this work is to optimize the performance of the Luenberger observer and integrate it with the aviation three-phase converter for the detection and control of human sports, achieving a major breakthrough. The present work can technically support the performance improvement of the Luenberger observer and facilitate the performance optimization of the aviation three-phase converter.

## 2. Research Theory and Methods

### 2.1. Three-Phase Converter

A converter is a device and circuit equipment converting the signal sent by the signal source for a particular purpose. At present, the converter has become the latest AC-AC variable frequency power supply. The converter generally has three control strategies: direct transformation method, indirect transformation method, and current tracking method [9]. The current tracking method compares the actual output current signal with the three-phase output current signal and determines the next working state according to the comparison results and the current switching state of the controlled element, that is, the switching operation task. It is characterized by easy adaptation, easy understanding, good robustness, and fast response [10]. Its disadvantages are the random distribution of harmonics, unstable switching frequency, unsatisfactory input current waveform, large waveform, etc. The indirect transformation method is also known as space vector modulation technology. Its main working principle is space vector transformation. In other words, AC-AC change becomes a virtual alternating current-direct current (AC-DC) conversion process, which can significantly improve the converter's performance. The implementation process needs a series of operations such as rectification and inverter [11]. It has a good effect on restraining low-order harmonics, but its specific working principle is complex and lacks the support of dynamic theoretical knowledge. The direct transformation method refers to the output of target voltage through the direct chopping process of input voltage, including scalar generation, harmonic injection method, coordinate transformation method, and equivalent conductance method [12].  Figure 1 reveals the main working principles of the three-phase converter.

As shown in Figure 1, the main working procedures of the converter include rectification, filtering, and inversion. Therefore, the principal working components of the converter are the rectifier, filter, and inverter. The primary function of the rectifier is to convert AC of a specific frequency and voltage into DC through a rectification procedure, which can be controllable or uncontrollable. The filter is mainly responsible for converting the pulsating DC output by the rectifier into a straight current through the filtering procedure. The filter can filter both DC and DC voltage [13]. The inverter is the central core of the conversion to convert the linear DC output by the filter into AC power through inversion and directly supplies the load current. However, its output AC voltage and frequency have nothing to do with the AC power supply input by the converter, so it is also called a passive inverter [14]. In summary, the three-phase converter plays a critical role in current control and contributes to improving current utilization efficiency.

### 2.2. Principle of the Luenberger Observer

The Luenberger observer adopts the methods of state estimation and state feedback in modern control theory. It uses measurable input and output variables to reconstruct the state that cannot be measured directly and carry out state feedback [15]. The state space of the linear system is described as follows:

(1) $$\begin{array}{c} \left\{\begin{array}{c} x=Ax+Bu\\ y=Cx \end{array}\right.. \end{array}$$

Here, *x* represents the state variable; *u* denotes the system input; *A* stands for the state matrix; *B* refers to the input matrix; and *C* denotes the output matrix.

Then, the state space description of the Luenberger observer can be written as follows:

(2) $$\begin{array}{c} \left\{\begin{array}{c} \hat{k}=A\hat{x}+Bu+H\left(y-\hat{y}\right)\\ \hat{y}=Cx \end{array}\right.. \end{array}$$

Here, $\hat{x}$ indicates the estimated value of the state variable, $\hat{y}$ signifies the estimated value of the output variable, and *H* refers to the feedback matrix [16].  Figure 2 reveals the basic principle of the Luenberger observer.

As shown in Figure 2, the characteristics of the controlled object can be detected through the Luenberger observer. Besides, the detected system of the Luenberger detector can be regulated according to the system feedback to improve the detection efficiency.

### 2.3. Structure of the Phase-Locked Loop

The basic three-phase phase-locked loop structure is based on the synchronous rotating coordinate system. The three-phase voltage **v**_**a**_, **v**_**b**_, and **v**_**c**_ are transformed into **v**_**d**_, **v**_**q**_, and **v**_**q**_ after a synchronous rotating coordinate transformation. The estimated value of the three-phase voltage phase angle *θ* is obtained after passing the voltage through the loop filter. Finally, the sine and cosine values of *θ* are calculated by a digital program or look-up table method [17]. The three-phase voltage can be expressed as follows:

(3) $$\begin{array}{c} \left\{\begin{array}{c} v_{a}=V_{s}\text{cos}\theta ,\\ v_{b}=V_{s}\text{cos}\left(\theta -\frac{2\pi }{3}\right)\\ v_{c}=V_{s}\text{cos}\left(\theta +\frac{2\pi }{3}\right) \end{array},\right. \end{array}$$

Here, **V**_**s**_ denotes the amplitude of the three-phase voltage, and *θ* represents the phase angle of the three-phase voltage. After the phase-locked loop is successfully phase-locked, **v**_**q**_ tends to 0. According to the synchronous rotation coordinate transformation, **v**_**q**_ can be approximately described as follows:

(4) $$\begin{array}{c} v_{q}=V_{s}sin\left(\theta -\theta \%\right)\approx V_{s}\left(\theta -\theta \%\right). \end{array}$$

The meaning of each parameter is the same as that in (3). As one of the power grid detection algorithms, the phase-locked loop algorithm plays an essential role in detecting the confidence of the amplitude, frequency, and phase of the single-phase and three-phase voltage positive sequence components [18]. It is also of great significance to the control strategy of the power converter. It is primarily responsible for detecting the frequency and phase of the grid voltage and controlling the output current of the power converter and the grid voltage synchronously. In addition, phase-locked loop technology is also the main technical principle of distributed generation systems, so it impacts the grid connection control performance of distributed generation systems [19].  Figure 3 displays the structural principle of the phase-locked loop technology.

As shown in Figure 3, the phase-locked loop technology can realize the control and transformation of the current and perform unified processing on the received signal to obtain a signal with the same frequency, dramatically reducing the error in the system operation. The phase value detected by the phase-locked loop technology is generally used during the working process to convert the three-phase coordinate system into a two-phase synchronous coordinate system. This operation converts the control current in the power grid from AC to DC, which provides appropriate methods for different use scenarios of current and improves the use efficiency of current [20].

### 2.4. Sensorless Vector Control

The sensorless vector control technology controls the excitation current and torque current through coordinate transformation processing, respectively. Then, the speed is identified to control the excitation current and torque current by controlling the voltage and current on the stator winding of the motor. This control method has a wide range of speed regulation, large starting torque, and reliable operation. However, the calculation is relatively complicated, and a special processor is generally required for calculation. Therefore, the real-time performance is not ideal, and the control accuracy is affected by the calculation accuracy.

The development of speed sensorless control technology begins with the conventional transmission control system with a speed sensor. The starting point of solving the problem is to use the detected stator voltage, current, and other easily detected physical quantities to estimate the speed to replace the speed sensor. The asynchronous motor vector control theory is used to solve the AC motor torque control problem. The basic principle of vector control is to measure and control the stator current vector of the asynchronous motor and control the excitation current and torque current of the asynchronous motor according to the principle of magnetic field orientation. It can achieve the purpose of controlling the torque of the asynchronous motor.

## 3. Design of the Phase-Locked Loop via Luenberger Observer

The study of (21) describes the relationship among the phase angle *θ* of the three-phase voltage, the angular frequency *ω*, and the derivative a of the angular frequency to time (the angular frequency is a linear transformation) [21].

(5) $$\begin{array}{c} \left\{\begin{array}{c} \theta =\omega t=a_{0}t^{2}+a_{0}t,\\ \omega =a_{0}t+\omega_{0},\\ a=a_{0}. \end{array}\right. \end{array}$$

In (21), **t** represents the time, *ω*_0_ denotes the initial value of *ω*, and **a**_0_ is a constant.

Then, the derivative of phase angle *θ* to time is

(6) $$\begin{array}{c} \omega^{\prime }=\frac{\mathrm{d\theta}}{\mathrm{dt}}=2a_{0}t+\omega_{0}. \end{array}$$

Then, the derivative of *ω*′ to time **a**′ is

(7) $$\begin{array}{c} a^{\prime }=\frac{\mathrm{da}\prime }{\mathrm{dt}}=2a_{0}. \end{array}$$

Based on equations (5–7), there is

(8) $$\begin{array}{c} \left\{\begin{array}{c} \omega =\frac{\omega^{\prime }+\sqrt{\omega^{\prime 2}-2\mathrm{\theta a}\prime }}{2}\\ a=\frac{a^{\prime }}{2} \end{array}\right.. \end{array}$$

The following equation defines a state space:

(9) $$\begin{array}{c} \left\{\begin{array}{c} x<Ax\\ y=Cx \end{array}\right.. \end{array}$$

There is

(10) $$\begin{array}{c} \begin{array}{c} x=\left[\begin{array}{c} \theta \\ \omega \\ a \end{array}\right]\ldots A=\left[\begin{array}{ccc} 0 & 1 & 0\\ 0 & 0 & 1\\ 0 & 0 & 0 \end{array}\right]\\ C=\left[\begin{array}{ccc} 1 & 0 & 0 \end{array}\right] \end{array}, \end{array}$$

According to (9), the Luenberger observer can be constructed as follows:

(11) $$\begin{array}{c} \left\{\begin{array}{c} \hat{x}=A\hat{x}+H\left(y-\hat{y}\right)\\ \hat{y}=C\hat{x} \end{array}\right.. \end{array}$$

Substituting (2) and (5) into (6), there are

(12) $$\begin{array}{c} \left[\begin{array}{c} \theta \\ \hat{\omega }\\ \hat{a} \end{array}\right]=\left[\begin{array}{c} \hat{\omega }\\ \hat{a}\\ 0 \end{array}\right]+H\left(\theta -\hat{\theta }\right)\approx \left[\begin{array}{c} \hat{\omega }\\ \hat{a}\\ 0 \end{array}\right]+H\frac{v_{q}}{V_{s}}=\left[\begin{array}{c} \hat{\omega }\\ \hat{a}\\ 0 \end{array}\right]+K_{q}=\left[\begin{array}{c} \hat{\omega }+k_{1}v_{q}\\ \hat{a}+k_{2}v_{q}\\ k_{3}v_{q} \end{array}\right], \end{array}$$

where

(13) $$\begin{array}{c} K=\frac{H}{V_{s}}=\left[\begin{array}{c} k_{1}\\ k_{2}\\ k_{3} \end{array}\right]. \end{array}$$

Then, the following equation holds according to (12):

(14) $$\begin{array}{c} \left\{\begin{array}{c} \hat{\theta }=\int \left(\hat{\omega }+k_{1}v_{q}\right)dt,\\ \hat{\omega }=\int \left(\hat{a}+k_{2}v_{q}\right)d,\\ \hat{a}=\int k_{3}v_{q}d \end{array}\right.. \end{array}$$

Then, the angular frequency $\hat{\omega }$ and the estimated sum of its derivative with respect to time $\hat{a}$ are

(15) $$\begin{array}{c} \left\{\begin{array}{c} \hat{\omega }=\frac{\hat{\omega }+\sqrt{{\hat{\omega }}^{\prime 2}-2\hat{\theta }\hat{a}\prime }}{2}\\ \hat{a}=\frac{a^{\prime }}{2} \end{array}\right.. \end{array}$$

The basic structure of the Luenberger observer phase-locked loop is determined through (15), as presented in Figure 4 [22].

The Luenberger observer phase-locked loop in Figure 4 is an optimized phase-locked loop technology based on the Luenberger observer. The combination of the Luenberger observer and the phase-locked loop technology improves the performance and efficiency of the Luenberger observer and reduces the probability of error.

## 4. Stability Analysis and Parameter Design of the Luenberger Observer Phase-Locked Loop

A small-signal model of the Luenberger observer phase-locked loop is established to collect main research data through real-time operation during the stability analysis and parameter design of the Luenberger observer phase-locked loop.  Figure 5 shows the small-signal model of the phase-locked loop of the Luenberger observer designed here [23].

In Figure 5, the small-signal model of the Luenberger observer phase-locked loop can improve the change efficiency and performance of the converter during current signal processing and conversion and reduce the overall error generation rate of the converter. The transfer function of the Luenberger observer phase-locked loop can be written as follows:

(16) $$\begin{array}{c} G_{1}\left(s\right)=\frac{\theta \prime \left(s\right)}{\left.\theta \phi_{s}\right)}=\frac{k_{1}s^{2}+k_{2}s+k_{3}}{s^{3}+k_{1}s^{2}+k_{2}s+k_{3}}. \end{array}$$

Under the premise of ensuring the stability of the Luenberger observer phase-locked loop, the poles of the transfer function are located in the left half-plane, which can be set as follows:

(17) $$\begin{array}{c} s_{0}=-w_{n}R,s_{1,2}=-w_{n}Exp\left(\pm j\phi \right), \end{array}$$

where **w**_**n**_ > 0, **R** >0, and 0 < *ϕ* < *π*/2. Substituting (17) into the characteristic equation of **G**(**s**), there is

(18) $$\begin{array}{c} k_{1}=\left(R+2cos\phi \right)w_{n}k_{2}=\left(1+2Rcos\phi \right)w_{n}^{2}k_{3}=Rw_{n}^{3}. \end{array}$$

Substitute (18) into (16) to get the following equation:

(19) $$\begin{array}{c} G\left(s\right)=\frac{\left(R+2cos\phi \right)w_{n}s^{2}+\left(1+2Rcos\phi \right)w_{n}^{2}s+Rw_{n}^{3}}{s^{3}+\left(R+2cos\phi \right)w_{n}s^{2}+\left(1+2Rcos\phi \right)w_{n}^{2}s+Rw_{n}^{3}}. \end{array}$$

The bandwidth **f**_**b**_ of the Luenberger Observer phase-locked loop is determined by the parameters **w**_**n**_, **R**, and *ϕ*. According to the definition of bandwidth, there is

(20) $$\begin{array}{c} 20lg\left|G\left(j2\pi f_{b}\right)\right|=20lg\left|G\left(j0\right)\right|-20lg\sqrt{2}. \end{array}$$

Then, the relationship between the bandwidth and each parameter can be expressed as follows:

(21) $$\begin{array}{c} \left[R^{2}w_{n}^{6}+\left(1+4R^{2}cos^{2}\phi -2R^{2}\right)w_{n}^{4}{\left(2\pi f_{b}\right)}^{2}\right.{\left.+\left(R^{2}+4cos^{2}\phi +2Rcos\phi -1\right)w_{n}^{2}{\left(2\pi f_{b}\right)}^{4}\right]}^{2}+{\left[Rw_{n}^{3}{\left(2\pi f_{b}\right)}^{3}-\left(R+2cos\phi \right)w_{n}{\left(2\pi f_{b}\right)}^{5}\right]}^{2}=\frac{1}{2}\left({\left[Rw_{n}^{3}-\left(R+2cos\phi \right)w_{n}{\left(2\pi f_{b}\right)}^{2}\right]}^{2}\right.{\left.+{\left[\left(1+2Rcos\phi \right)w_{n}^{2}\left(2\pi f_{b}\right)-{\left(2\pi f_{b}\right)}^{3}\right]}^{2}\right)}^{2}. \end{array}$$

The correlation between **w**_**n**_ and **f**_**b**_, **R**, and **f**_**b**_, and *ϕ* and **f**_**b**_ can be defined according to (21).

## 5. Sensorless Vector Control

Sensorless vector control methods are primarily divided into the direct calculation method, flux linkage position estimation method, high-frequency injection method, synovial observer method, and extended Kalman filter method [24]. First, the direct calculation method obtains the motor's voltage and flux linkage equation according to the mathematical model of the permanent magnet synchronous motor to calculate the required angle and speed of the motor directly. The flux linkage position estimation method estimates the rotor position and speed of the motor by calculating the specific position of the back EMF. Generally, the position of the back EMF is determined by the space vector position of the stator flux linkage. Under a certain current, the rotor vector position and flux linkage vector position of the permanent magnet synchronous motor can be calculated. Therefore, the space vector position of the flux linkage can be determined through the motor voltage and current to locate the vector position of the rotor at the current time. The high-frequency signal injection method uses the protruding machine effect of the motor to add high-frequency signals to the motor's stator windings and then demodulates the rotor position and speed information of the motor after the corresponding filter [25]. The injected high-frequency signal is generally divided into high-frequency current and high-frequency voltage signals. This algorithm is less sensitive to motor parameters and can obtain the motor rotor position and speed at zero and low speeds. The synovial observer can change the control loop of the state observer into a synovial variable structure. Its discontinuity is the biggest difference from other control methods. With the change of time, the system structure will also change, so the system will move under certain characteristics with time, called a synovial movement, also known as sliding mode [26]. This algorithm has strong robustness due to its outstanding adaptability to motor parameters. The advantage of the extended Kalman filter method is that it can obtain real-time observation signals from random noise signals. However, the precision standard of processor chips and related devices is extremely high to meet the control requirements of this algorithm, dramatically increasing the hardware cost. This algorithm is relatively complex, resulting in a considerable calculation amount in the system operation [27]. Therefore, it is essential to delve into vector control. This work studies the phase-locked loop combined with the optimization of vector control to improve the application efficiency of the Luenberger observer.

## 6. Structure and the Small-Signal Model of the Phase-Locked Loop Based on Steady-State Linear Kalman Filter

The discrete-domain third-order prediction model of the steady-state linear Kalman filter phase-locked loop based on the grid phase angle *θ*, angular frequency *ω*, and the derivative *α* of the angular frequency to time can be expressed as follows [28]:

(22) $$\begin{array}{c} x_{n}=Dx_{n-1}\\ y_{n}=Cx_{n}\\ x=\left[\begin{array}{c} \theta \\ \omega \\ \omega \end{array}\right]D=\left[\begin{array}{ccc} 1 & T & \frac{T^{2}}{2}\\ 0 & 1 & T\\ 0 & 0 & 1 \end{array}\right]\\ C=\left[\begin{array}{ccc} 1 & 0 & 0 \end{array}\right]. \end{array}$$

where **n** denotes the sampling coefficient and **T** refers to the sampling period.

According to (17), the phase-locked loop of the steady-state linear Kalman filter is designed through the following two steps:

(1) Predict the sampling state at the next moment:
  (23) $$\begin{array}{c} x_{n}=D{\hat{x}}_{n-1}. \end{array}$$
(2) Correct the predicted state by the phase angle error:

(24) $$\begin{array}{c} {\hat{x}}_{n}=x_{n}+ge_{n}. \end{array}$$

In (24), $g={\left[\begin{array}{c} g_{1},g_{2},g_{3} \end{array}\right]}^{T}$, and **e**_**n**_ ≈ *θ*_**n**_ − *θ*_**n**_^%^.

Figure 6 displays the structure of the phase-locked loop of the steady-state linear Kalman filter.

According to Figure 6, using the steady-state linear Kalman filter can optimally estimate the system state through the system input and output observation data. Since the observation data includes the influence of noise and interference in the system, the optimal estimation can also be regarded as a filtering process. Data filtering is a data processing technique that removes noise and restores real data. However, the steady-state linear Kalman filter phase-locked loop model in Figure 6 is excessively complicated, so this structure needs to be simplified to reduce the workload of the system without damaging its working ability. Therefore, the above steady-state linear Kalman filter phase-locked loop model is designed to simplify to optimize its system.  Figure 7 indicates the small-signal model of the phase-locked loop of the steady-state linear Kalman filter.

The study of (25) demonstrates the transfer function **G**_2_(**s**) of the linear Kalman filter.

(25) $$\begin{array}{c} G_{2}\left(s\right)=\frac{\theta \left(s\right)}{\theta \left(\rho_{s}\right)}=\frac{g_{1}^{\prime }s^{2}+g_{2}^{\prime }s+g_{3}^{\prime }}{s^{3}+g_{1}^{\prime }s^{2}+g_{2}s+g_{3}^{\prime }}. \end{array}$$

It can be seen that the Luenberger observer phase-locked loop and the linear Kalman filter phase-locked loop have the same transfer function of the small-signal model.

However, the phase-locked loop of the Luenberger observer is simpler than that of the linear Kalman filter phase-locked loop in algorithm design, which only needs one equation (29). Moreover, the phase-locked loop of the linear Kalman filter does not have the function of frequency locking.

The study of (26) denotes the state space equation of the continuous domain of (22).

(26) $$\begin{array}{c} \frac{\mathrm{dx}}{\mathrm{dt}}=\frac{x_{n}-x_{n-1}}{T}. \end{array}$$

Then, there are

(27) $$\begin{array}{c} x_{n}=\mathrm{Ax}, \end{array}$$

(28) $$\begin{array}{c} y=\mathrm{Cx}, \end{array}$$

(29) $$\begin{array}{c} x=\left[\begin{array}{c} \theta \\ \omega \\ a \end{array}\right]A=\left[\begin{array}{c} 0,1,0\\ 0,0,1\\ 0,0,0 \end{array}\right], \end{array}$$

(30) $$\begin{array}{c} C=\left[\begin{array}{c} 1,0,0 \end{array}\right]. \end{array}$$

The angular frequency output by the phase-locked loop of the steady-state linear Kalman filter is not the actual angular frequency of the power grid. Therefore, it does not have the function of frequency locking.

## 7. Application Research of the Luenberger Observer

### 7.1. Application of the Luenberger Observer in the Phase-Locked Loop

The Luenberger Observer phase-locked loop and the Linear Kalman Filter phase-locked loop are simulated in the Matlab/Simulink environment for performance comparison. The three-phase voltage is expressed as (3). According to (21), the relationship between **w**_**n**_ and **f**_**b**_ when **R**=1 and *ϕ*=*π*/3, the relationship between **R** and **f**_**b**_ when **w**_**n**_=1 and *ϕ*=*π*/3, and the relationship between *ϕ* and **f**_**b**_ when **R**=1 and **w**_**n**_=1 are also calculable.  Figure 8 shows the specific relationship between the above elements.

As shown in Figure 8, under given **R** and **w**_**n**_, the change of *ϕ* has few effects on **f**_**b**_. Besides, when **f**_**b**_ is larger than 0.5 Hz, the change of **w**_**n**_ has a greater influence on **f**_**b**_ than that of **R**. Therefore, the appropriate bandwidth **f**_**b**_ of the Luenberger observer phase-locked loop is selected when **R**=1 and *ϕ*=*π*/3, and **w**_**n**_ can be determined accordingly. First, it is essential to compare the phase-locking performance of the two phase-locked loops under the condition of grid voltage and frequency sudden change. The grid voltage frequency is set to change from 360 Hz to 800 Hz at 0.11 s abruptly. The performance of the two phase-locked loops with a bandwidth of 50 Hz and 100 Hz is compared. The parameter design methods of the two phase-locked loops are the same because the transfer functions of the small-signal models of the two phase-locked loops are the same. According to (19), **w**_**n**_  = 110.964, *R* = 1, and *ϕ* = *π*/3; **w**_**n**_  = 221.928, *R* = 1, and *ϕ* = *π*/3. According to (18), **k**_1_  = *g*1´ = 221.928, **k**_2_  = *g*2´ = 24626.019, and **k**_3_  = *g*3´ = 1366300.764; **k**_1_  = *g*1´ = 443.857, **k**_2_  = *g*2´ = 98504.074, and **k**_3_  = *g*3´ = 10930406.108.  Figure 9 reveals the results of the output phase angle of the two phase-locked loops under the condition of grid voltage and frequency sudden change.

According to Figure 9, the two phase-locked loops have the same phase-locking effect under the same bandwidth because the transfer functions of the small-signal models of the two phase-locked loops are the same. When the voltage frequency of the three-phase power supply changes, the angular frequency of the output of the two phase-locked loops will change to some extent under the 50 Hz and 100 Hz bandwidths.  Figure 10 shows the specific results of the output angle frequency under the change of the angle frequency and voltage frequency of the three-phase power supply.

As shown in Figure 10, when the power supply voltage frequency changes linearly, the output angular frequency of the Luenberger observer phase-locked loop can be consistent with the power supply voltage angular frequency under both bandwidths. On the contrary, there is a particular gap between the output angular frequency and the power supply voltage angular frequency of the steady-state linear Kalman filter phase-locked loop. This result proves that the Luenberger observer phase-locked loop has the function of frequency locking.

### 7.2. Application Research on Sensorless Vector Control

The optimization of sensorless vector control can significantly improve the performance of the Luenberger observer. Therefore, this work optimizes the Luenberger vector control method through the phase-locked loop and compares it with the traditional Luenberger vector control. The comparison of control angles can intuitively show the specific optimization results.  Figure 11 provides the comparison result.

As shown in Figure 11, by comparing the control angles before and after optimization, it can be found that the vector control angle of the Luenberger observer is closer to the mechanical angle, reducing the control error.  Figure 12 provides the comparison results of the control angle error before and after optimization.

Figure 12 suggests that the control angle of the Luenberger observer has been dramatically improved after vector control optimization. In the error comparison before and after optimization, the maximum error angle before the optimization is about 0.24°, while the maximum error result after optimization is about 0.18°. It can be seen that the vector control has been dramatically improved. The experimental result provides an essential reference for improving the comprehensive use efficiency of the Luenberger observer. In summary, this work has carried out a comprehensive optimization of the Luenberger observer and a relatively complete evaluation of the application of the aviation three-phase converter. Compared with the research of Cheng and Li (2022), the research reported here optimizes the Luenberger observer and aeronautical three-wire converter while designing their conditions in practical applications, which are suitable for practical applications [30].

## 8. Conclusion

This work is a comprehensive study of the Luenberger observer phase-locked loop and the three-phase variation vector control method in aviation. The optimization of the Luenberger observer system, combined with the comprehensive application of the phase-locked loop technology in the three-phase converter that receives the aviation variable frequency power supply, can effectively improve the efficiency and conversion function. In this way, the Luenberger observer can be applied to the detection of sports performance to offer a reference for improving sports efficiency. The Luenberger observer phase-locked loop is compared with the steady-state linear Kalman filter PLL phase-locked loop. It is found that the two phase-locked loops have the same small-signal model transfer function, so they have the same phase-locked effect at the same bandwidth. However, the design algorithm of the Luenberger observer phase-locked loop is simpler than that of the stationary linear Kalman filter phase-locked loop. In addition, when the angular frequency of the input supply voltage varies linearly, the Luenberger Observer phase-locked loop has a frequency-locking function that the steady-state linear Kalman filter phase-locked loop lacks. Finally, the vector control method of the aviation converter is optimized. The combination of the vector control method and the phase-locked loop technology can effectively improve the control efficiency of the Luenberger observer. The performance comparison demonstrates that the unoptimized Luenberger observer has a significant deviation in the control angle. In contrast, the control angle deviation of the Luenberger observer is significantly reduced after optimization. The control angle error before the optimization is about 0.24°, while the control angle error of the optimized Luenberger observer is about 0.18°. It can be seen that the Luenberger observer reported here has achieved breakthrough results. Although this work studied the vector control method of the Luenberger observer, its comprehensive optimization is not mature enough and deserves further research in the future.

## Figures and Tables

**Figure 1:** Basic working principle of the converter. (a) The working circuit; (b) the working flow.

**Figure 2:** Working rationale of the Luenberger observer.

**Figure 3:** Structural principle of the phase-locked loop.

**Figure 4:** Structure of the Luenberger observer phase-locked loop.

**Figure 5:** Small-signal model of the Luenberger observer phase-locked loop.

**Figure 6:** Structure of the phase-locked loop of the steady-state linear Kalman filter. (a) The discrete domain; (b) the continuous domain.

**Figure 7:** Small signal model of the phase-locked loop of the steady-state linear Kalman filter.

**Figure 8:** Relationship between **f**_**b**_ and **w**_**n**_, **R**, and *ϕ*.

**Figure 9:** Output phase angle of two kinds of phase-locked loops under the sudden change of power supply voltage frequency. (a) Under the bandwidth of 50 Hz; (b) under the bandwidth of 100 Hz.

**Figure 10:** Output angular frequency of two phase-locked loops under the linear transformation of power supply voltage and frequency. (a) Under the bandwidth of 50 Hz; (b) under the bandwidth of 100 Hz.

**Figure 11:** Comparison results of the control angle of the Luenberger vector before and after optimization. (a) Before optimization; (b) after optimization.

**Figure 12:** Comparison of the vector control error before and after the optimization.

## Data Availability

The data used to support the study are included in the paper.
